The article "Synergistic Antibiofilm Effect of Thymol and Piperine in Combination with Aminoglycosides Antibiotics against Four Salmonella enterica Serovars" was published in 2021. Journal: Evid Based Complement Alternat Med.

# Synergistic Antibiofilm Effect of Thymol and Piperine in Combination with Aminoglycosides Antibiotics against Four *Salmonella enterica* Serovars

**DOI:** 10.1155/2021/1567017

**Published:** 2021-10-27

**Authors:** Christian Ramsès Tokam Kuaté, Borel Bisso Ndezo, Jean Paul Dzoyem

**Affiliations:** Laboratory of Microbiology and Antimicrobial Substances, Department of Biochemistry, Faculty of Science, University of Dschang, Dschang, Cameroon

## Abstract

Biofilms related to human infection have high levels of pathogenicity due to their resistance to antimicrobial agents. The discovery of antibiofilm agents is necessary. One approach to overcome this problem is the use of antibiotics agents' combination. This study aimed to determine the efficacy of the combination of natural products thymol and piperine with three aminoglycosides antibiotics, amikacin, kanamycin, and streptomycin against biofilm-forming *Salmonella enterica.* The microtiter plate assay method was used to evaluate the biofilm-producing capacity of the isolates. Minimum inhibitory concentration (MIC) and minimum bactericidal concentration were determined by the broth microdilution method. The inhibition of biofilm formation and biofilm eradication was determined using the microtiter broth method. The checkerboard method was used to determine the combined effects of natural products with aminoglycosides antibiotics. All the tested isolates showed various levels of biofilm formation. Overall, combinations provided 43.3% of synergy in preventing the biofilm formation and 40% of synergy in eradicating preformed biofilms, and in both cases, no antagonism was observed. The combination of thymol with kanamycin showed a synergistic effect with 16- to 32-fold decrease of the minimum biofilm eradication concentration (MBEC) of kanamycin. The interaction of piperine with amikacin and streptomycin also revealed a synergistic effect with 16-fold reduction of the minimum biofilm inhibitory concentration (MBIC). The combination of thymol with the three antibiotics showed a strong synergistic effect in both inhibiting the biofilm formation and eradicating the preformed biofilm. This study demonstrates that thymol and piperine potentiate the antibiofilm activity of amikacin, kanamycin, and streptomycin. These combinations are a promising approach therapeutic to overcome the problem of *Salmonella enterica* biofilm-associated infections. In addition, these combinations could help reduce the concentration of individual components, thereby minimizing the nephrotoxicity of aminoglycosides antibiotics.

## 1. Introduction

The effectiveness of several antibacterial agents is currently decreasing due to the emergence of multidrug-resistant pathogens, which represent a serious challenge to medicine and healthcare [1, 2]. One of the main causes of resistance is the formation of biofilms [3]. Bacterial biofilm is defined as an association of bacterial cells, fixed to surfaces, abiotic or biotic surfaces, which are embedded in a complex extracellular matrix of polymeric substances (EPS). EPS has a varying chemical composition, mainly composed of polysaccharides, glycoproteins, and phospholipids. The composition and amount of the components of the extracellular matrix are different depending on the bacterial species. The EPS extremely increases microbial resistance, by preventing the passage of antibiotics and other harmful substances into the bacterial community [4]. In addition, biofilms formed by bacteria are more resistant to antimicrobials than free-living microorganisms, with minimum eradication concentrations 10 to 1000 times higher than in planktonic bacteria [5]. *Salmonella* spp. are Gram-negative facultative intracellular anaerobes that cause a wide spectrum of diseases named salmonellosis. Most of the human pathogenic *Salmonella* serovars belong to the *enterica* subspecies. These serogroups include *Salmonella*Typhi, *Salmonella* Enteritidis, *Salmonella* Paratyphi, *Salmonella* Typhimurium, and *Salmonella* Choleraesuis [6]. Human salmonellosis generally manifests two kinds of disorders: typhoid fever caused by typhoidal *Salmonella enterica* serotypes such as *Salmonella* Typhi, and another is gastroenteritis caused by nontyphoidal *Salmonella* serotypes such as *Salmonella* Enteritidis [7]. Worldwide estimates of nontyphoidal Salmonella range from 200 million to 1.3 billion, with an estimated death toll of 3 million each year. The serovars responsible for typhoid or enteric fever, typhi, and paratyphi that cause systemic illness lead to an estimated 22 million cases and 216,000 deaths worldwide, and the International Vaccine Institute estimated that there were 11.9 million cases of typhoid fever and 129,000 deaths in low- to middle-income countries in 2010 [8]. Several reports document that the production of biofilm exerts a key role in supporting the colonization and chronic persistence of *Salmonella* spp. in the body [9]. The biofilm formation is also contributed to *Salmonella* virulence, since bacteria in the biofilm are more resistant to antibiotics and host immune system, resulting in chronic infection and the development of *Salmonella* carrier state [10]. Therefore, it is important to search for alternative therapeutics to control biofilm-associated *Salmonella* infections.

The article "Synergistic Antibiofilm Effect of Thymol and Piperine in Combination with Aminoglycosides Antibiotics against Four Salmonella enterica Serovars" was published in 2021. Journal: Evid Based Complement Alternat Med.

Aminoglycosides are potent and broad-spectrum antibiotics used against bacterial infections. Their primary mechanism of action relates to inhibition of bacterial protein synthesis via binding to bacterial 30S ribosomal subunit through hydrogen bond and ionic interactions [11]. However, despite their broad-spectrum activity, nephrotoxicity and ototoxicity of aminoglycosides have been major adverse effects that limit their clinical use [12]. Fluoroquinolones still remain the main therapeutic drugs of choice for the treatment of life-threatening salmonellosis and typhoid fever in most African countries with poor resources, but with treatment failures due to multidrug-resistant strains [13]. Aminoglycoside antibiotic agents are mainly used for the treatment of extracellular pathogen infections, such as *Pseudomonas aeruginosa* and *Escherichia coli* infections, and thus are not commonly used for the treatment of typhoid fever [14]. However, the lack of new antibiotics necessitates the improvement of existing ones. Many reports suggest that the use of drug combinations against resistant bacterial pathogens has better efficacy compared to monotherapy, as the use of a single agent is highly associated with the occurrence of resistance [15]. The combination of aminoglycosides with other antibiotics has been shown to enhance their bactericidal activity [16]. In addition, a recent study reported that potentiating aminoglycoside antibiotics can reduce their toxic side effects [17].

Plant-derived compounds have been widely used to combat microbial infections, because they are inexpensive and easy to extract [18]. They have effective antibacterial properties against both Gram-positive and Gram-negative bacteria. Since these phytochemicals are known to modulate or modify resistance mechanisms in bacteria, their potential use in combinations with antibiotics can help potentiate the activity of the western drugs, resulting in increased efficacy [19]. Several studies have proposed that natural compounds in combination with antibiotics are a new strategy for developing therapies for infections caused by bacterial species and that natural plant products can potentiate the activity of antibiotics in combination [20]. Thymol is a major constituent in the essential oil of the thyme plant; it is known to have various biological properties such as antibacterial, antifungal, antioxidant, and cognitive-enhancing activities [21]. Thymol inhibits bacterial growth by altering the membrane permeability and disturbing both protein synthesis and binary fission. Piperine, a naturally occurring alkaloid, is the major bioactive component responsible for the pungency of commonly consumed spices black pepper (*Piper nigrum*), white pepper, and long pepper (*Piper longum*). At subinhibitory concentrations, both thymol and piperine reduce biofilm formation [22, 23]. Few studies reported the interaction of thymol and piperine with antibiotics. In this regard, we undertook this study to investigate the *in vitro* antibiofilm activity of thymol and piperine in combination with three aminoglycosides antibiotics, amikacin, kanamycin, and streptomycin, against biofilm formation by four *S. enterica* serovars including *S*. Typhi, *S*. Typhimurium, *S*. Enteritidis, and *S*. Choleraesuis.

The article "Synergistic Antibiofilm Effect of Thymol and Piperine in Combination with Aminoglycosides Antibiotics against Four Salmonella enterica Serovars" was published in 2021. Journal: Evid Based Complement Alternat Med.

## 2. Materials and Methods

### 2.1. Microorganisms and Growth Conditions

The reference strain *S.* Typhi (ATCC 6539) used in the present study was purchased from American Type Culture Collection (ATCC). Clinical isolates, *S.* Enteritidis, *S.* Typhi, *S*. Typhimurium, and *S.* Choleraesuis, were provided by “*Centre Pasteur du Cameroun*.” All bacterial strains were plated from cultures, which were stored at − 80°C onto *Salmonella-Shigella* agar (SSA) (Condalab) for 18–24 h at 37°C. Cultures were subsequently subcultured and maintained on Muller Hinton agar (MHA Sigma-Aldrich) plates at 4°C until needed for further bioassay.

### 2.2. Chemical and Natural Products

Amikacin disulfate salt and streptomycin sulfate (Acros Organics) and kanamycin sulfate (Thermo Scientific), as well as thymol and piperine, were purchased from Sigma-Aldrich. Dimethyl sulfoxide (DMSO), p-iodonitrotetrazolium chloride (INT), and 3-(4,5-dimethylthiazole-2-yl)-2,5-diphenyltetrazolium bromide (MTT) were also purchased from Sigma-Aldrich. SSA and MHB media were purchased from Dominique Dutscher SAS, France.

### 2.3. Antimicrobial Susceptibility Tests

The activities of natural products and aminoglycosides against planktonic cells were evaluated by determining minimum inhibitory concentration (MICs) and minimum bactericidal concentration (MBCs). The broth microdilution method as previously described was used [24, 25]. The MBC/MIC ratio was then calculated to determine the bactericidal (MBC/MIC ≤4) or bacteriostatic (MBC/MIC ˂4) effect [26].

### 2.4. Ability Biofilm Formation

The microtiter plate assay method was used to quantitatively determine biofilm production by a microplate reader, as described by Kirmusaoğlu and Kasiki, with some modifications [27]. In brief, 100 *µ*L of MHB supplemented with 2% glucose and 100 *µ*L of bacterial inoculum (1.5 × 10^6^ CFU/mL) were introduced into 96-well flat-bottomed sterile polystyrene microplate. Then, the microplate was incubated at 37°C for 6 h, 12 h, 24 h, 48 h, and 72 h. After incubation, planktonic cells in the well of the microplate were discharged by washing twice with 300 *µ*L of phosphate-buffered saline (PBS) at 7.2 pH. To perform biofilm formation, MTT reduction assay was used. Briefly, 200 *μ*L of MTT (0.5 mg/mL) prepared in PBS was introduced into each well, and the microplate incubated at 37°C for 4 hours. Uninoculated wells containing sterile MHB supplemented with 2% glucose were considered to be negative controls and were used as blanks. After incubation, MTT solution was aspirated, and 150 *μ*L of DMSO was introduced, and the microplate was measured spectrophotometrically at 570 nm by a microplate reader.

The article "Synergistic Antibiofilm Effect of Thymol and Piperine in Combination with Aminoglycosides Antibiotics against Four Salmonella enterica Serovars" was published in 2021. Journal: Evid Based Complement Alternat Med.

### 2.5. Antibiofilm Assays

#### 2.5.1. Biofilm Inhibition Assay

The inhibition of biofilm by thymol and piperine and aminoglycosides was carried out according to the protocol described by Ahmed et al., with slight modifications [28]. Briefly, 100 *µ*L of bacterial inoculum (1.5 × 10^6^ CFU/mL) and 100 *µ*L of concentration of antibiotics or natural products were introduced in the microplate. Final concentrations of antibiotics and natural products respectively range from 0.25 to 512 *µ*g/mL and 2 to 4096 *µ*g/mL. Then, the microplate was incubated at 37°C for 4 h. After incubation, the plates were gently emptied, washed three times with a phosphate buffer solution at pH 7.2, and treated as described for the biofilm formation assay mentioned above. Wells containing bacteria and MHB supplemented glucose 2% were used as the positive control, while wells containing MHB supplemented glucose 2% without bacteria were used as the negative control. The percentage inhibition of metabolic activity was calculated as follows:

(1) $$\begin{array}{c} \%\text{Inhibition metabolic activity}=\frac{\left({\text{OD}}_{\text{control}}-{\text{OD}}_{\text{blanc}}\right)-\left({\text{OD}}_{\text{test}}-{\text{OD}}_{\text{blanc}}\right)}{\left({\text{OD}}_{\text{control}}-{\text{OD}}_{\text{blanc}}\right)}\times 100. \end{array}$$

The minimal biofilm inhibitory concentration (MBIC) was defined as the lowest concentration of aminoglycosides and natural products required to inhibit the formation of biofilm, which inhibits 100% of metabolic activity.

#### 2.5.2. Biofilm Eradication Assay

The determination of biofilm eradication by thymol, piperine, and antibiotics was performed through cell viability in the preformed biofilm [27]. Briefly, 200 *µ*L of bacterial inoculum (7.5 × 10^5^ CFU/mL) was introduced into the microplate and incubated at 37°C for 48 h. After it had formed, the microplates were gently emptied and washed three times with PBS. Then, 100 *µ*L of MHB supplemented with 2% glucose and 100 *µ*L of aminoglycosides or natural products at concentrations ranging from 0.5 to 1024 *µ*g/mL and 2–4096 *µ*g/mL, respectively, were added into the wells. After 24 h incubation at 37°C, the medium was removed, and the plates were washed three times with PBS. The microplate was treated as described for the biofilm inhibition assay mentioned above. Bioassay was performed in triplicate and repeated three times. The percentage eradication of metabolic activity was calculated as previously described, and the minimal biofilm eradication concentration (MBEC) was recorded as the lowest concentration of aminoglycosides or natural products, which reduces 100% of metabolic activity.

The article "Synergistic Antibiofilm Effect of Thymol and Piperine in Combination with Aminoglycosides Antibiotics against Four Salmonella enterica Serovars" was published in 2021. Journal: Evid Based Complement Alternat Med.

### 2.6. Combination Studies

#### 2.6.1. Combination of Aminoglycosides with Thymol and Piperine to Prevent Biofilm Formation

Checkerboard assay was used for the determination of the combined effects of aminoglycosides whit thymol or piperine to prevent biofilm formation. The method was used according to the technique described by Cokol et al., with some modifications [29]. Briefly, 50 *µ*L of Mueller-Hinton broth supplemented with 2% glucose was distributed into each well of microdilution plates. The antibiotic of the combination was serially diluted along the abscissa, and natural products were serially diluted along the ordinate. 100 *µ*L of bacterial inoculum (1.5 × 10^6^ CFU/mL) was added to each well, and the plates were incubated at 37°C for 24 h under aerobic conditions. Final concentration ranges from 0.125 to 128 *µ*g/mL for antibiotics, 16–1024 *µg*/mL for piperine, and 8–512 *µ*g/mL for thymol. After incubation, the plates were gently emptied and washed three times with a phosphate buffer solution at pH 7.2. The well containing bacteria and MHB supplemented with 2% glucose was used as a positive control, while the well containing MHB without bacteria was used as blank. MTT reduction assay as described above was used to perform the metabolic activity in the biofilm. The lowest minimum biofilm inhibitory concentration (MBIC) of antibiotics or natural products that inhibited metabolic activity in biofilm was determined as described above. The fractional inhibitory concentration index (FICI) was used to perform the effect of combination and calculated as follows: FICI = (MBIC of antibiotic in the combination/MBIC of antibiotic alone) + (MBIC of natural product in the combination/MBIC of natural products alone). FICI was interpreted as follows: synergy when FICI ≤0.5, additivity when 0.5 ˂ FICI ≤ 1, indifference when 1 ˂ FICI ≤ 4, and antagonism when FICI ˃4 [30].

#### 2.6.2. Combination of Aminoglycosides with Thymol and Piperine against Preformed Biofilm

Checkerboard was also used as previously described. After biofilm formation for 48 h, the plate was gently emptied and washed three times with PBS. Then, 50 *µ*L of antibiotic and 50 *µ*L of natural products were introduced into the plate as described above, and 100 *µ*L of MHB supplemented with 2% glucose was introduced to the plate. The final concentration ranges from 0.125 to 128 *µ*g/mL for antibiotics and 16–1024 *µ*g/mL for piperine and thymol.

The article "Synergistic Antibiofilm Effect of Thymol and Piperine in Combination with Aminoglycosides Antibiotics against Four Salmonella enterica Serovars" was published in 2021. Journal: Evid Based Complement Alternat Med.

After incubation at 37°C for 24 h, the medium was gently removed, and the plate was washed three times with PBS. At the end of incubation, the MTT reduction assay described above was assessed to evaluate the metabolic activity of biofilm, and minimum biofilm eradication concentration MBEC was determined. To perform the effect of the combination, the FICI was calculated and interpreted as described above.

### 2.7. Statistical Analysis

All tests were considered significant at *p* < 0.05 using the software GraphPad Prism 8.0. Results were presented as means ± standard deviation from three replicates of experiments. The difference between mean values was determined by the analysis of variance (ANOVA). The analysis was performed by Fisher's least significant difference.

## 3. Results

### 3.1. Antimicrobial Susceptibility Test

The test of the sensitivity of the bacterial to aminoglycosides and natural products (MIC and MBC in *µ*g/mL) is consigned in Table 1. MIC ranged from 1 to 4 *µ*g/mL for amikacin and streptomycin, and from 2 to 4 *µ*g/mL for kanamycin. The MBC of amikacin and streptomycin ranged from 4 to 16 *µ*g/mL, and from 8 to 16 *µ*g/mL for kanamycin. With thymol, MIC ranged from 64 to 128 *µ*g/mL, and MBC from 128 to 256 *µ*g/mL. On different strains, the MIC values of piperine were 512 or 1024 *µ*g/mL, and MBC for all isolates was >1024 *µ*g/mL. Thymol was bactericidal to all *Salmonella enterica* with MBC/MIC ratio <4.

### 3.2. Kinetics of Biofilm Formation

The kinetics of the four *Salmonella enterica* serovars biofilm growth was performed at 6 h, 12 h, 24 h, 48 h, and 72 h of incubation. The absorbance at 570 nm was plotted against these different times (Figure 1). From the kinetics analyses, a gradual increase was observed in biofilm formation up to 48 h. At 72 h, the biofilm formation of all isolates compared to 48 h dropped. At 48 h of incubation, *S.* Choleraesuis (OD = 2.08) and *S.* Typhimurium (OD = 1.87) were the best biofilm-forming isolates. However, after 72 h incubation, the biofilm formation decreased with the OD values from 2.08 to 1.31 for *S.* Choleraesuis and from 1.87 to 1.53 for *S.* Typhimurium.

### 3.3. Antibiofilm Effect of Aminoglycosides Antibiotics and Natural Products Alone

The MBIC and MBEC of aminoglycosides (amikacin, kanamycin, and streptomycin), thymol, and piperine alone were determined. Then, their interactions were appreciated by determining FICI. The results are presented in Table 2. The MBIC values ranged from 4 to 8 *µ*g/mL for amikacin, from 8 to 16 *µ*g/mL for kanamycin, and from 4 to 16 *µ*g/mL for streptomycin. The MBIC values of amikacin and streptomycin were 2–8 times higher than their MIC for each antibiotic. Additionally, MBIC values of kanamycin were 2–16 times higher than the MIC ones. For thymol and piperine, the MBIC values ranges were 256–1024 *µ*g/mL and 1024 *µ*g/mL, respectively.

The article "Synergistic Antibiofilm Effect of Thymol and Piperine in Combination with Aminoglycosides Antibiotics against Four Salmonella enterica Serovars" was published in 2021. Journal: Evid Based Complement Alternat Med.

### 3.4. Effect of the Combination of Aminoglycosides Antibiotics with Natural Products against the Biofilm Formation

The result of the combination of natural products with aminoglycosides antibiotics against biofilm formation is presented in Table 2. Combination of amikacin with thymol decreased the MBIC value of amikacin from 4 to 8 *µ*g/mL to 0.5–1 *µ*g/mL with synergy effect (FICI = 0.09–0.31) against all *Salmonella enterica* isolates. A synergistic effect was obtained in the combination of kanamycin with thymol against all *Salmonella enterica* serovars tested, decreasing 8 to 32 times their MBIC values. The combination of streptomycin with thymol showed a synergy effect against *S.*Choleraesuis with a 32-fold reduction of the MBIC of streptomycin. The assessment of the interaction between piperine-amikacin revealed a synergetic effect against *S.* Typhimurium and *S.* Choleraesuis with, respectively, 16-fold and 8-fold reduction of the MBIC of amikacin. The synergy effect was also obtained in the combination of kanamycin with piperine against *S.*Typhi ATCC 6539 and *S.*Choleraesuis with a 4-fold reduction of the MBIC value of kanamycin.

### 3.5. Effect of the Combination Aminoglycosides Antibiotics with Natural Products against the Preformed Biofilm

The results of the capacity of thymol, piperine, and aminoglycosides to destroy preformed biofilm by the four *Salmonella enterica* serovars are shown in Table 3. The MBEC values of amikacin and kanamycin ranged from 64 to 128 *µ*g/mL, while MBEC of streptomycin ranged from 128 to 256 *µ*g/mL. For thymol, MBEC ranged from 512 to 1024 *µ*g/mL on all *Salmonella enterica* serovars, while MBEC values of piperine were 1024 *µ*g/mL. The interaction of natural products with aminoglycosides antibiotics was also determined against the preformed biofilm of the four *Salmonella enterica* serovars, and the results are also found in Table 3. Synergism was observed in the interaction of thymol-amikacin against all *Salmonella enterica* serovars except *S.* Typhi ATCC 6539, reducing the MBEC value of amikacin by 16 to 64 times with the FICI values in the range of 0.13 to 0.31. A ratio of 3/5 synergy was obtained in the combination of thymol with kanamycin and decreasing 16–32 times the MBEC of kanamycin. The biofilm eradication potency of piperine in combination with amikacin showed only one synergistic effect against *S.* Choleraesuis (FICI = 0.16) with a 16 times reduction of the MBEC of amikacin, whereas the interaction of piperine-kanamycin and piperine-streptomycin decreased, 8- to 16-fold, the MBEC of each antibiotic. The combination of amikacin with piperine allowed to obtain a synergistic effect only against *S.* Choleraesuis (FICI = 0.16) reducing the MBEC value from 64 to 2 *µ*g/mL.

The article "Synergistic Antibiofilm Effect of Thymol and Piperine in Combination with Aminoglycosides Antibiotics against Four Salmonella enterica Serovars" was published in 2021. Journal: Evid Based Complement Alternat Med.

## 4. Discussion

The steadily increasing bacterial resistance to existing antimicrobial drugs is a serious problem, and therefore, there is a need to search for new approaches to antibacterial resistance especially by biofilm formation. The aminoglycoside antibiotics are not recommended for treating enteric fever due to infection with *Salmonella enterica* serovar. However, the lack of new antibiotics and the urgent need to search for new antibiotic agents necessitate the improvement of other existing ones. The use of antibiotics alone sometimes does not produce effective action. To overcome this problem, a combination of drugs is often used. Therefore, we reasoned that natural adjuvant that potentiates the activity of aminoglycoside could be a strategy to rescue these antibiotics. Moreover, some aminoglycoside antibiotics such as gentamicin and amikacin have been found to be effective against multidrug resistant *S. enterica* serovar Typhi infection in vitro. In this study, the combination of three aminoglycosides antibiotics (amikacin, kanamycin, and streptomycin) with two bioactive natural products (thymol and piperine) was investigated against four biofilm-forming *Salmonella enterica* serovars including *S*. Typhi, *S*. Typhimurium, *S*. Enteritidis, and *S*. Choleraesuis.

As expected, in preliminary experiments, the antibacterial effect performed against planktonic cells showed that all the four *Salmonella enterica* serovars were sensitive to the three aminoglycosides antibiotics tested. However, the antibacterial activity of thymol and piperine was less effective compared to antibiotics. The antibacterial activity of natural products has been categorized as very good when MIC ≤15 µg/mL, good when 15 < MIC ≤ 25 *µ*g/mL, moderate when 25 < MIC ≤ 100 *µ*g/mL, and low when MIC > 100 *µ*g/mL [31]. On this basis, Thymol was more effective than piperine. Thymol presented moderate activity against *S.* Typhi ATCC 6539, S. Enteritidis, and *S.*Typhi, while piperine showed low antibacterial activity against all *S. enterica* serovars tested. These results are in agreement with the literature since, in a previous study, thymol was reported as the most effective essential oil against twelve *Salmonella* Typhimurium strains with the lowest MICs values ranging from 32 to 128 *μ*g/mL [32]. Furthermore, the disruption of membrane integrity was shown to be the antibacterial mechanism of action of thymol against *Salmonella* Typhimurium [33]. Piperine derivatives having pyridine scaffold were synthesized by Amperayani et al. and observed that they exhibit antimicrobial activity when tested against a range of microbial pathogens including *Salmonella* Typhi [34]. Piperine is the major plant alkaloid present in black pepper (*Piper nigrum*) and long pepper (*Piper longum*), and the black pepper is used as a traditional medicine for its antibacterial activity. Black pepper is reported to possess antibacterial activity and biological activities and pungency of pepper are due to the presence of piperine [35].

The article "Synergistic Antibiofilm Effect of Thymol and Piperine in Combination with Aminoglycosides Antibiotics against Four Salmonella enterica Serovars" was published in 2021. Journal: Evid Based Complement Alternat Med.

In this study, the biofilm formation capacity of the four *Salmonella enterica* serovars was assessed. The kinetic study of biofilm formation revealed an increase of the biofilm formation up to 48 h, followed by a drop at 72 h. Therefore, the best time for biofilm formation was 48 h. These findings follow the known biofilm formation steps [36], and the increase observed of the biofilm formation from 6 to 48 h indicates the attachment and maturation phases, while the drop at 72 h corresponds to the dispersal phase.

The three aminoglycosides antibiotics and the two bioactive natural products showed the ability both to prevent the biofilm formation and to disperse the preformed biofilm. As expected, the MBIC and MBIC values of the tested compounds were higher than their respective MIC values.

This was an expected finding since the biofilm formation, which is also a mechanism of virulence, is well known as one of the mechanisms of resistance used by bacteria [37]. The biofilms formed by bacteria are generally more resistant to antimicrobials than planktonic microorganisms, with minimum eradication concentrations 10 to 1000 times higher than those in planktonic bacteria [5]. Thymol was shown to induce a great reduction, about 4-log, at 624 *μ*g/mL against mature *Salmonella* Enteritidis biofilm [38].

Piperine was reported to have bioavailability-enhancing activity for some nutritional substances and some drugs [39]. Therefore, we also assessed the antibiofilm effect of piperine as well as thymol in association with the three aminoglycosides antibiotics. Overall, these combinations provided 43.3% of synergy in preventing the biofilm formation and 40% of synergy in eradicating preformed biofilms, and in both cases, no antagonism was observed. The association of phytochemicals with the conventional drug was shown to be more effective in combating bacteria biofilm and synergistic effects resulting from the combination of antibiotics with different plant extracts and derived compounds have been studied by several researchers [40]. Liu et al. reported a synergistic effect of four components of essential oil including thymol combined with streptomycin on planktonic and biofilm-associated *Salmonella* Typhimurium [41]. To the best of our knowledge, this is the first study reporting a synergistic antibiofilm efficacy of piperine with antibiotics against biofilms bacterial pathogens.

The article "Synergistic Antibiofilm Effect of Thymol and Piperine in Combination with Aminoglycosides Antibiotics against Four Salmonella enterica Serovars" was published in 2021. Journal: Evid Based Complement Alternat Med.

These promising results allowed us to confirm the synergistic effects between the natural products and the three aminoglycosides antibiotics studied. The data obtained show a significant reduction in the concentrations of antibiotics when used in association either with thymol or piperine. In particular, this work emphasizes the efficacy of thymol or piperine in enhancing the activity of antibiotics. Moreover, our results underlined the large reduction of the quantities of individual components employed in the combination giving the antibiofilm synergy concerning the quantity used alone to inhibit the biofilm.

## 5. Conclusion

From this study, it appears that thymol and piperine act synergically in combination with amikacin, streptomycin, and kanamycin on biofilm-associated *Salmonella enterica.* These synergistic interactions may help in designing a more potent, safe, and effective novel antibiofilm agent against typhoid fever and gastroenteritis caused by nontyphoidal *Salmonella enterica*. Besides, this combination could also help reduce the concentration of individual components, thereby minimizing the known nephrotoxicity and ototoxicity of aminoglycosides antibiotics.

## Figures and Tables

**Figure 1:** Kinetics of the biofilm-producing capacity of four *Salmonella enterica* serovars. Data represent means ± SD (error bars) of three experiments. Values marked with the same letter do not differ significantly (*p* < 0.05 according to Fisher's least significant difference).

**Table 1:** MIC and MBC of thymol, piperine, and antibiotics against planktonic cells of four *Salmonella enterica* serovars.

Isolates	Susceptibility (*µ*g/mL)	Natural products		Antibiotics		
		Thymol	Piperine	Amikacin	Kanamycin	Streptomycin
*S.* Typhi *ATCC 6539*	MIC	64	512	2	4	2
	MBC	256	>1024	4	16	4
	R	4	>2	2	4	2
*S.* Enteritidis	MIC	64	1024	1	4	1
	MBC	128	>1024	4	16	4
	R	2	>1	4	4	4
*S.* Typhi	MIC	64	1024	1	4	1
	MBC	256	>1024	8	16	4
	R	4	>1	8	4	4
*S.* Typhimurium	MIC	128	512	2	4	1
	MBC	128	>1024	4	8	4
	R	1	>2	2	2	4
*S.* Choleraesuis	MIC	128	512	4	2	4
	MBC	256	>1024	16	8	16
	R	2	>2	4	4	4

MIC: minimum inhibitory concentration, MBC: minimum bactericidal concentration, R: MBC/MIC ratio.

The article "Synergistic Antibiofilm Effect of Thymol and Piperine in Combination with Aminoglycosides Antibiotics against Four Salmonella enterica Serovars" was published in 2021. Journal: Evid Based Complement Alternat Med.

**Table 2:** Minimum biofilm inhibitory concentration (MBIC) and effects of the combination of thymol/piperine with amikacin, kanamycin, and streptomycin against biofilm formation of four *Salmonella enterica* serovars.

Isolates	Antibiotics	MBIC (*µ*g/mL)							MBIC reduction fold (antibiotic)		FICI/INT	
		Alone			Combined							
		ATB	Thy	Pip	ATB/Thy	Thy	ATB/Pip	Pip	ATB/Thy	ATB/Pip	ATB/Thy	ATB/Pip
*S.* Typhi ATCC 6539	Amikacin	8	256	1024	0.5	32	1	512	16	8	0.19/S	0.63/Ad
	Kanamycin	8	256	1024	1	64	2	128	8	4	0.38/S	0.38/S
	Streptomycin	8	256	1024	0.5	256	2	1024	16	4	1.06/I	1.25/I
*S.* Enteritidis	Amikacin	8	1024	1024	0.25	64	0.5	512	32	16	0.09/S	0.56/Ad
	Kanamycin	8	1024	1024	8	256	2	512	1	4	1.25/I	0.75/Ad
	Streptomycin	4	1024	1024	0.5	512	0.25	256	8	16	0.63/Ad	0.31/S
*S.* Typhi	Amikacin	4	256	1024	0.25	64	1	512	16	4	0.31/S	0.75/Ad
	Kanamycin	8	256	1024	2	128	1	1024	4	8	0.75/Ad	1.13/I
	Streptomycin	16	256	1024	8	64	4	1024	2	4	0.75/Ad	1.25/I
*S*. Typhimurium	Amikacin	8	256	1024	1	8	0.5	256	8	16	0.16/S	0.31/S
	Kanamycin	8	256	1024	0.5	16	1	1024	16	8	0.13/S	1.13/I
	Streptomycin	8	256	1024	8	64	0.5	512	1	16	1.25/I	0.56/Ad
*S.* Choleraesuis	Amikacin	8	256	1024	0.25	64	1	256	32	8	0.28/S	0.38/S
	Kanamycin	16	256	1024	2	256	4	128	8	4	1.13/I	0.38/S
	Streptomycin	8	256	1024	0.25	64	1	512	32	8	0.28/S	0.63/Ad

MBIC: minimum biofilm inhibitory concentration, Thy: thymol, Pip: piperine, ATB/Thy: combination of antibiotic with thymol, ATB/Pip: combination of antibiotic with piperine, FICI: fractional inhibitory concentration index, INT: interpretation, S: synergy, Ad: additivity, I: indifference.

**Table 3:** Minimum biofilm eradication concentration (MBEC) and effects of the combination of thymol/piperine with amikacin, kanamycin, and streptomycin against preformed biofilm of four *Salmonella enterica* serovars.

Isolates	Antibiotics	MBEC (*µ*g/mL)							MBEC reduction fold (antibiotic)		FICI/INT	
		Alone			Combined							
		ATB	Thy	Pip	ATB/Thy	Thy	ATB/Pip	Pip	ATB/Thy	ATB/Pip	ATB/Thy	ATB/Pip
*S.* Typhi ATCC 6539	Amikacin	128	512	1024	8	256	4	1024	16	64	0.56/Ad	1.03/I
	Kanamycin	128	512	1024	4	128	16	256	32	8	0.28/S	0.38/S
	Streptomycin	128	512	1024	64	128	8	1024	2	16	0.75/Ad	1.06/I
*S.* Enteritidis	Amikacin	128	1024	1024	2	256	8	512	64	16	0.27/S	0.56/Ad
	Kanamycin	64	1024	1024	4	256	8	512	16	8	0.31/S	0.63/Ad
	Streptomycin	128	1024	1024	16	1024	8	1024	8	16	1.13/I	1.06/I
*S.* Typhi	Amikacin	128	512	1024	8	32	16	512	16	8	0.13/S	0.63/Ad
	Kanamycin	128	512	1024	8	256	8	1024	16	16	0.56/Ad	1.06/I
	Streptomycin	256	512	1024	16	512	16	256	16	16	1.06/I	0.31/S
*S*. Typhimurium	Amikacin	64	512	1024	4	128	8	512	16	8	0.31/S	0.63/Ad
	Kanamycin	128	512	1024	8	128	8	128	16	16	0.31/S	0.19/S
	Streptomycin	128	512	1024	16	256	16	256	8	8	0.63/Ad	0.38/S
*S.* Choleraesuis	Amikacin	64	512	1024	1	128	2	128	64	16	0.27/S	0.16/S
	Kanamycin	64	512	1024	4	512	4	512	16	16	1.06/I	0.56/Ad
	Streptomycin	256	512	1024	16	256	32	512	16	8	0.56/Ad	0.63/Ad

MBEC: minimum biofilm eradication concentration, Thy: thymol, Pip: piperine, ATB/Thy: combination of antibiotic with thymol, ATB/Pip: combination of antibiotic with piperine, FICI: fractional inhibitory concentration index, INT: interpretation, S: synergy, Ad: additivity, I: indifference.

The article "Synergistic Antibiofilm Effect of Thymol and Piperine in Combination with Aminoglycosides Antibiotics against Four Salmonella enterica Serovars" was published in 2021. Journal: Evid Based Complement Alternat Med.

## Data Availability

The data used to support the findings of this study are available upon reasonable request from the corresponding author.
